The article "Pleiotropic role of Drosophila phosphoribosyl pyrophosphate synthetase in autophagy and lysosome homeostasis" was retracted in 2022. Reasons: errors in the data; errors in the results or conclusions.

# Pleiotropic role of Drosophila *phosphoribosyl pyrophosphate synthetase* in autophagy and lysosome homeostasis

**DOI:** 10.1371/journal.pgen.1008376

**Published:** 2019-09-05

**Authors:** Keemo Delos Santos, Minhee Kim, Christine Yergeau, Steve Jean, Nam-Sung Moon

**Affiliations:** 1 Department of Biology, Developmental Biology Research Initiative, McGill University, Montreal, Quebec, Canada; 2 Faculté de Médecine et des Sciences de la Santé, Département d’Anatomie et de Biologie Cellulaire, Université de Sherbrooke, Sherbrooke, QC, Canada; Stanford University School of Medicine, UNITED STATES

## Abstract

Phosphoribosyl pyrophosphate synthetase (PRPS) is a rate-limiting enzyme whose function is important for the biosynthesis of purines, pyrimidines, and pyridines. Importantly, while missense mutations of *PRPS1* have been identified in neurological disorders such as Arts syndrome, how they contribute to neuropathogenesis is still unclear. We identified the Drosophila ortholog of *PRPS* (*dPRPS*) as a direct target of RB/E2F in Drosophila, a vital cell cycle regulator, and engineered *dPRPS* alleles carrying patient-derived mutations. Interestingly, while they are able to develop normally, *dPRPS* mutant flies have a shortened lifespan and locomotive defects, common phenotypes associated with neurodegeneration. Careful analysis of the fat body revealed that patient-derived PRPS mutations result in profound defects in lipolysis, macroautophagy, and lysosome function. Significantly, we show evidence that the nervous system of *dPRPS* mutant flies is affected by these defects. Overall, we uncovered an unexpected link between nucleotide metabolism and autophagy/lysosome function, providing a possible mechanism by which PRPS-dysfunction contributes to neurological disorders.

## Author summary

Phosphoribosyl pyrophosphate synthetase (PRPS) is an important enzyme in nucleotide synthesis: the building blocks of DNA and RNA and other important metabolites. Importantly, while PRPS is mutated in neurological disorders such as Arts syndrome, Charcot-Marie-Tooth disease, and nonsyndromic sensorineural deafness, it is currently unclear why PRPS dysfunction leads to neurological disorders. In this study, we engineered a *Drosophila* model of ARTS syndrome and discovered that PRPS mutations result in defects in lysosome-mediated and autophagy processes, which are known to be important for neuronal homeostasis. Our study provides crucial insights into the way that PRPS mutations contribute to neurological disorders.

## Introduction

Phosphoribosyl pyrophosphate synthetase (PRPS) is a rate-limiting enzyme in the biosynthesis of purine, pyrimidine, and, pyridine nucleotides (Fig 1A). Purine and pyrimidine nucleotides are the building blocks of RNA and DNA while pyridine nucleotides, such as NAD^+^ and NADP, are important co-factors in many enzymatic reactions. PRPS produces phosphoribosyl pyrophosphate (PRPP), a common precursor of the five-carbon sugar subunit of nucleotides [1]. The essential role of PRPS in nucleotide metabolism is illustrated through its conservation among all free-living organisms, ranging from *E*.*coli* to humans.

**Fig 1:** *phosphoribosyl pyrophosphate synthetase* (*PRPS*) is a RBF1- and Capicua-regulated gene. (A) Schematic describing the role of PRPS in nucleotide biosynthesis is shown. PRPS converts ribose-5-phosphate from the pentose phosphate pathway into phosphoribosyl pyrophosphate (PRPP), which is required for the synthesis of various nucleotides such as purines, pyrimidines and pyridines. (B) Somatic clones of *cic*^*Q474X*^ mutant cells are generated in third instar larval eye imaginal discs. *cic* mutant clones are marked by the lack of βGal signal (red). A GFP protein trap allele of *dPRPS* (green, see materials and methods and S1B Fig), is used to monitor expression of dPRPS in control and *cic* mutant clones. A magnified view of the indicated area (white box) is also presented. Outlined in yellow denote the border between wild type and *cic* mutant clones. Scale bar: 100 μm for white and 30 μm for yellow. (C) Somatic clones of cells carrying *rbf1*^*cas21*^ mutations are generated in eye imaginal discs. Anti-RBF1 is used to visualize *rbf1* mutant cells and the same GFP trap allele described in B is used to monitor dPRPS expression. Scale bar: 100 μm for white and 30 μm for magnified view. (D) Levels of *dPRPS* transcript were measured by qRT-PCR from control eye discs (oreR) and eye discs entirely composed of *rbf1*^*cas21*^ (three biological replicates; mean values ± Standard Error of the Mean (SEM) are expressed relative to levels in control). (E) Levels of *dPRPS* transcript were measured by qRT-PCR from control eye discs (*yw*) and eye discs entirely composed of *cic*^*Q474X*^ (three biological replicates; mean values ± SEM are expressed relative to levels in control). (F) Chromatin immunoprecipitation assays are used to determine dE2F1 and RBF1 binding sites in the *dPRPS* promoter. The arrows in the diagram indicate the location of P1 and P3 primer pairs. *rnrS* is a well-established dE2F1 and RBF1 target gene and *Actin* is used as a negative control. Percentage enrichment relative to the input is calculated based on three independent triplicated experiments. Values represent the mean of triplicated biological replicates and error bars represent standard deviation. Statistical testing in 1D-E were performed using two-tailed t-tests where * = p ≤ 0.05.

In humans, three *PRPS* orthologs exists. Notably, *PRPS1* mutations were identified in a number of X-linked neurological disorders: Arts syndrome, Charcot-Marie-Tooth disease (CMT), and nonsyndromic sensorineural deafness [2, 3]. All *PRPS1* mutations identified from patients are missense mutations affecting enzymatic activity to varying degrees. Arts syndrome is the most severe form of *PRPS1* disease, and is characterized by infant death, sensorineural hearing loss, intellectual disability, hypotonia, and ataxia. The fact that no nonsense mutations were identified suggests that *PRPS1* is essential for embryonic development and patients with missense mutations retain a certain level of PRPS1 function. Knockout mutants of PRPS orthologs have been generated in a number of animal models. *PRPS1* knockout mice were generated as a part of a high-throughput screening of mouse genes important for skeletal muscle development [4]. Not surprisingly, *PRPS1* was identified as an X-linked gene required for animal viability, supporting the notion that the gene is essential for embryonic development. In contrast, *PRPS2* knockout mice are viable and fertile with no discernable developmental defects. This suggests that other mouse *PRPS* orthologs, *PRPS1* and *PRPS1L1*, can compensate for the loss of *PRPS2* [5]. Interestingly, while *PRPS2* is non-essential for development, *PRPS2* knockout mice are resistant to *Eμ–Myc*-driven cancer development, suggesting that *PRPS2* is specifically required for tumorigenesis [5]. A zebrafish model of PRPS deficiency has also been recently generated [6]. The mutant animals of the two zebrafish PRPS orthologs, *PRPS1a* and *PRPS1b*, fail to properly develop and show some phenotypic similarities to human PRPS1-associated diseases. Notably, only null alleles of *PRPS* were generated in both mouse and zebrafish models and the biological consequence of patient-derived *PRPS1* mutations have not been directly examined.

Retinoblastoma (RB) family proteins are evolutionarily conserved regulators of the cell cycle [7, 8]. They are best known for their ability to control S-phase entry by directly binding and regulating E2F family transcription factors. Cell cycle-dependent phosphorylation of RB ensures the timely activation of E2F, whose target genes are required for proper cell cycle progression [8]. Notably, RB is also involved in other cellular processes including cell metabolism [9]. For instance, studies in RB mutant flies and mice have shown that the loss of RB alters glutamate catabolism to compensate for an increased demand for DNA synthesis [9, 10]. Moreover, a recent study using a proteomics appoach demonstrated that RB inactivation profoundly affects protein levels that are associated with mitochondrial function [11]. While theses studies clearly demonstrated metabolic reprogramming in RB-deficient cells, genes and pathways that are crucial for these changes are yet to be determined.

Studies in mammals suggest that PRPS activity is regulated by signals that control cellular growth. In addition to being regulated by Myc [5], the enzymatic activity of PRPS is regulated by 5′ AMP-activated protein kinase (AMPK) [12]. The hexameric form of PRPS, the active configuration of the enzyme, is converted to inactive monomers by AMPK phosphorylation. This study demonstrated that AMPK, which senses energy stress, directly regulates the rate of nucleotide synthesis by controlling PRPS activity. Interestingly, a recent study in Drosophila using DNA adenine methyltransferase identification (DamID) technique identified *CG6767*, which codes the only Drosophila *PRPS* (*dPRPS*), as one of the Capicua (Cic) targets [13]. Cic is a transcriptional repressor downstream of the EGFR/Ras pathway, which our lab previously identified as an important determinant of proliferation and survival of *rbf1* mutant cells, a Drosophila ortholog of RB [14]. In addition, the *CG6767* locus was identified as a locus occupied by a Drosophila E2F, dE2F1, in S2 cells [15]. Given its rate-limiting function in nucleotide metabolism and possible role downstream of RBF1/dE2F1, we sought to investigate the *in vivo* function of dPRPS. Since dPRPS has 89% protein sequence identity with the mammalian PRPS1 (S1A Fig) and the *in vivo* consequence of the patient-derived mutations has not been directly tested, we generated *dPRPS* alleles that carry mutations identified from Arts syndrome, *dPRPS*^*Q165P*^ and *dPRPS*^*R228W*^ [2, 16]. Interestingly, while these flies are viable and fertile, they are highly sensitive to nutrient deprivation. We discovered that their susceptibility to starvation is in part caused by failure to mobilize their lipid reserves due to profound defects in autophagy and lysosome function. Further analysis also revealed that *dPRPS*^*Q165P*^ and *dPRPS*^*R228W*^ have defects during cellular response to oxidative stress and accumulate lipid droplets and protein aggregates in the brain. Our findings revealed an unexpected link between nucleotide metabolism and autophagy/lysosome function and provide a possible explanation by which PRPS1 dysfunction results in neurological disorders.

## Results

### *dPRPS* is a direct target of RBF1/dE2F1

We first tested if *dPRPS* expression is indeed regulated by Cic and RBF1. For this task, we used a protein trap allele of *dPRPS*, wherein a GFP coding sequence is inserted in-frame at the N-terminal region of the protein (S1B Fig). Comparing the expression of *GFP-trap* in eye imaginal discs containing *cic* mutant clones confirmed that dPRPS expression is normally repressed by Cic (Fig 1B). In addition, a similar experiment in eye imaginal discs containing *rbf1* mutant clones also showed that RBF1 normally represses *dPRPS* expression (Fig 1C). RT-qPCR using RNA isolated from eye imaginal discs mostly composed of mutant cells of *cic* and *rbf1* further demonstrated that *dPRPS* expression is indeed regulated by Cic and RBF1 (Fig 1D and 1E). We also confirmed that *dPRPS* is a direct RBF1/dE2F1 target by chromatin immunoprecipitation (ChIP), which showed a recruitment of RBF1 and dE2F1 to the promoter region of *CG6767* (Fig 1F). Taken together, our results demonstrate that *dPRPS* is a Cic- and RBF1-regulated gene and suggest that PRPS may link nucleotide metabolism to the rate of proliferation.

### Patient-derived *dPRPS* mutations prevent a Ras-induced hyperplasia and result in reduced longevity and locomotion

*Mi09951* is a publicly available insertional *dPRPS* allele that disrupts splicing between the exon 1 and 2 of *dPRPS* and places a polyadenylation site in the intron (S1B Fig). As a consequence, the expression of *dPRPS* exons downstream of exon 1 is severely disrupted in *Mi09951* (S1C Fig). Trans-heterozygous between a deficiency line covering the *dPRPS* locus and the *Mi09951* or *GFP-Trap* allele resulted in early larval lethality (S1D Fig), making them difficult to analyze. Therefore, to better understand the *in vivo* function of PRPS and to directly assess the physiological consequence of patient-derived mutations, we engineered two *dPRPS* alleles that carry the mutations identified from Arts syndrome via CRISPR/Cas9: *dPRPS*^*Q165P*^ and *dPRPS*^*R228W*^ (S2A Fig and Fig 2A). These patient-derived mutations did not largely affect dPRPS transcript levels (S2B Fig) and unlike *Mi09951* or *GFP-Trap* mutants, *dPRPS*^*Q165P*^ and *dPRPS*^*R228W*^ flies are viable and fertile with no discernable developmental defects. In addition, developmental timing of *dPRPS*^*Q165P*^ and *dPRPS*^*R228W*^ is not affected and the size of wings and eyes of adult flies are normal (S2C–S2E Fig). However, enzymatic function of dPRPS is compromised in both mutants, validated by measuring the relative ATP levels in control and *dPRPS* mutant adult flies (Fig 2B). Compromised dPRPS function in *dPRPS*^*Q165P*^ and *dPRPS*^*R228W*^ flies was further demonstrated by their ability to suppress a Ras-induced phenotype. Since Cic is a crucial factor in regulating proliferation downstream of the EGFR/Ras pathway, we reasoned that dPRPS activity may be required for the Ras-induced tumor phenotype. To test this hypothesis, both mutations were introduced to a genetic background overexpressing an activated form of Ras (Ras^V12^) in the eye, which results in a characteristic hyperplastic overgrowth [17]. Strikingly, the Ras^V12^-induced phenotype is strongly suppressed in the *dPRPS*^*Q165P*^ or *dPRPS*^*R228W*^ mutant background, indicating that dPRPS is required for Ras-induced hyperplastic overgrowth (Fig 2C). Molecular markers such as phospho-Histone H3 and cleaved caspase revealed that dPRPS is required by Ras^V12^ to overcome developmentally-regulated cell cycle arrest and apoptosis (S2F and S2G Fig). Overall, these results demonstrate that *dPRPS*^*Q165P*^ and *dPRPS*^*R228W*^ are hypomorphic alleles of *dPRPS* that maintain a sufficient amount of PRPS function to support animal development.

**Fig 2:** Patient-derived *dPRPS* mutations prevent a Ras-induced hyperplasia and result in reduced longevity and locomotion. (A) The diagram shows the locations of patient-derived missense mutations introduced to the *dPRPS* genes via CRISPR/Cas9 system (*dPRPS*^*Q165P*^ *and dPRPS*^*R228W*^; see materials and methods and S2A Fig). (B) The graph shows the relative ATP levels in control and *dPRPS*^*Q165P*^ and *dPRPS*^*R228W*^ adult females. Error bar indicate SEM from triplicated experiments (n = 5 per experiment). (C) Scanning Electron Microscopy (SEM) images of adult eyes showing the effect of overexpressing an activated form of Ras (*Ras*^*V12*^) in control (left panel), *dPRPS*^*Q165P*^ (middle panel) and *dPRPS*^*R228W*^ (right panel) eyes are shown. Scale bar: 200 μm. (D) *dPRPS*^*Q165P*^ and *dPRPS*^*R228W*^ flies show reduced lifespan than control. Error bar indicate SEM from triplicated three independent experiments (n = 100 per experiment). (E) Climbing ability of *dPRPS*^*Q165P*^, *dPRPS*^*R228W*^ flies and control flies were measured at day 3 and day 30. Error bar indicate SEM from triplicated three independent experiments (n = 200 per experiment). Statistical testing in 2B was performed using One-way ANOVA where ns = p>0.05; ** = p ≤ 0.01; *** = p ≤ 0.001. Statistical testing in 2D were performed using log-rank test where * = p ≤ 0.05. Statistical testing in 2E were performed using One-way ANOVA comparison to control at endpoint (t = 120 sec), p<0.0001; * = p ≤ 0.05; ** = p ≤ 0.01.

Because the mutant alleles are derived from Arts syndrome, we examined whether *dPRPS*^*Q165P*^ and *dPRPS*^*R228W*^ adult flies display any signs of neurological defects. Supporting the notion that dPRPS is important for the nervous system, a recent study identified *CG6767* as a gene required for proper olfactory behaviour [18]. Consistent with other fly models of neurodegenerative disorders that have a shortened lifespan [19], both patient-derived PRPS mutations demonstrate reduced lifespan. The lifespan of control versus *dPRPS* mutant flies were compared and at 50 days after eclosion, approximately 25% of *dPRPS*^*Q165P*^ and *dPRPS*^*R228W*^ flies survived while more than 50% of control flies were still alive (Fig 2D). In addition, climbing tests were performed to examine locomotive and nervous system function [20]. Strikingly, *dPRPS*^*Q165P*^ and *dPRPS*^*R228W*^ flies display locomotive defects as early as three days after eclosion. While most control flies were able to reach a target line by 50 seconds, only about 75–80% of *dPRPS* mutants were able to climb to the threshold (Fig 2E left panel). In addition, at 30 days after eclosion, a significant fraction of *dPRPS* mutant flies were unable to reach the target line while most control flies were able to do so in two minutes (Fig 2E right panel). Overall, patient-derived mutations compromise *dPRPS* function and produce phenotypes associated with neurological defects.

### *dPRPS* mutants have lipid mobilization defects

The Drosophila fat body functions as an energy reserve in the form of lipid droplets and plays a role similar to the mammalian liver and adipose tissue [21]. Interestingly, publicly available expression data from microarrays and RNA-sequencing analyses indicate that *dPRPS* is highly expressed in the Drosophila fat body (S3A Fig). This was confirmed by the *GFP-trap* allele that showed strong expression in the fat body (S3B Fig). Because animal survival during starvation is tightly linked to fat usage [21], we examined the sensitivity of d*PRPS*^*Q165P*^ and *dPRPS*^*R228W*^ adult flies to starvation. Indeed, upon complete nutrition withdrawal, *dPRPS*^*Q165P*^ and *dPRPS*^*R228W*^ flies die about two days faster than age-matched control flies (S3C Fig). We next visualized the lipid droplets in the fat body during the progression of starvation. While the size of lipid droplets decreases in control flies, it remains relatively unchanged in *dPRPS*^*Q165P*^ and *dPRPS*^*R228W*^ flies (Fig 3A and 3B). Additionally, quantification of triglyceride (TAG) levels, the primary lipid form in which the fat is stored, revealed a similar trend wherein TAG levels are significantly reduced in the control flies during starvation but are relatively unchanged in the *dPRPS* mutants (Fig 3C). This observation suggests that the increased sensitivity to starvation in *dPRPS*^*Q165P*^ and *dPRPS*^*R228W*^ flies may be caused by failure to use their lipid reserves. To test this hypothesis, we overexpressed *Lipase 4* (*Lip4*), a lipase used in starvation-mediated lipolysis [22], in control and *dPRPS* mutant fat bodies using *lsp2-Gal4* (Fig 3D). *Lip4* overexpression had little to no effect on the survival of control flies during starvation. However, *Lip4* overexpression in *dPRPS*^*Q165P*^ and *dPRPS*^*R228W*^ flies significantly improved their survival, suggesting that defects in lipid mobilization contribute to their hypersensitivity to nutrient withdrawal.

**Fig 3:** *dPRPS* mutants have starvation-induced lipid mobilization defects. (A) Adult fat bodies from control and *dPRPS* mutant flies under fed (left panel) and starved (right panel) conditions are stained with 4′,6-diamidino-2-phenylindole (DAPI, blue) and LipidTOX (red) to visualize nuclei and lipid droplets, respectively. Scale bar: 100 μm. (B) A graph showing the average size of lipid droplets in control, *dPRPS*^*Q165P*^ and *dPRPS*^*R228W*^ flies at indicated time points during starvation is presented. Error bar indicate SEM from triplicated three independent experiments (n = 150 per experiment). Statistical testing was performed using One-way ANOVA comparison to control at endpoint (t = 48 hours), p<0.1291, where ** = p ≤ 0.01. (C) A graph showing normalized triacylglycerol (TAG) levels in control and *dPRPS* mutant adult flies during starvation is presented. Error bar indicate SEM from triplicated three independent experiments (n = 5 per experiment). Statistical testing was performed using One-way ANOVA comparison to control at endpoint (t = 48 hours), p = 0.0283, where * = p ≤ 0.05; ** = p ≤ 0.01. (D) A graph showing the survival of control and *dPRPS* mutant adult flies under starvation is presented. The effect of expressing a lipase under the control of a fat body-specific driver, *lsp2-Gal4*, is also included in the graph (*Lps2Gal4>UAS-lipase*). Error bar indicate SEM from triplicated three independent experiments (n = 25 per experiment). Statistical significance was measured using Log-Rank test as compared to control (*Lsp2Gal4;Control*). p≤0.01 *Lsp2Gal4;Q165P*, p≤0.01 *Lsp2Gal4;R228W*, p≥0.05 *Lsp2Gal4>UAS-lipase; Control*, p ≤ 0.05 *Lsp2Gal4>UAS-lipase;Q165P*, p ≤ 0.05 *Lsp2Gal4>UAS-lipase; R228W*.

### *dPRPS* is required for starvation-induced autophagy

During starvation, autophagy is one of the primary mechanisms to mobilize lipids [23]. Intracellular lipids are sequestered in double membrane vesicles called autophagosomes and delivered to the lysosome for their eventual degradation for energy production and macromolecular synthesis [24, 25]. To determine whether autophagy is deregulated in *dPRPS* mutants, we expressed GFP-Atg8a, a molecular marker of autophagy, in the fat body [26]. In control flies, GFP-Atg8a signals under fed condition show low number of basal puncta that increase with starvation (Fig 4A). Strikingly, in *dPRPS* mutant flies, not only are the basal GFP-Atg8a signals lower than the control, but the number of GFP-Atg8a puncta induced by starvation does not increase to the level observed in the control flies under fed condition (Fig 4A lower panel). Fundamental defects in autophagy under fed condition was further demonstrated by abnormal accumulation of Ref(2)p/p62, which is normally turned over by autophagy [27]. Even under normal growth conditions, Ref(2)p/p62 puncta were readily observed in *dPRPS*^*Q165P*^ fat bodies, while being largely absent in control flies (Fig 4B), supporting the notion that basal autophagy is deregulated in *dPRPS* mutant flies. To functionally confirm the autophagy defect revealed by the molecular markers, we examined the effect of depleting core autophagy proteins *atg8a* and *atg16* in *dPRPS* fat bodies [26, 28]. We reasoned that *atg8a* or *atg16* depletion should have minimal effects in *dPRPS* mutant flies if autophagy is already compromised. Indeed, while *atg8a* or *atg16* knockdown decreases the survival rate of control flies upon starvation, it has no significant effect on the survival of *dPRPS* mutant flies (Fig 4C and 4D). Overall, these data suggest that dPRPS dysfunction caused by patient-derived mutations affects autophagy and may explain why *dPRPS* mutants are unable to breakdown lipid droplets during starvation.

**Fig 4:** dPRPS is required for starvation-induced autophagy. (A) GFP-tagged Atg8a (GFP-Atg8a, green) was expressed via *lsp2-Gal4* to monitor autophagy under fed (upper panels) and starved (lower panels) conditions in adult fat bodies of control and *dPRPS* mutants. DAPI is used to visualize nuclei (blue). Magnified views of the indicated area (white box) is also presented in the right. Scale bar 100 μm. Graphs show quantification of GFP-Atg8a signals (GFP puncta per nuclei) under fed and starved conditions. Error bar indicate SEM from triplicated three independent experiments (n = 125 per experiment). (B) Adult fat bodies of control and *dPRPS* mutant fat bodies stained with an anti-Ref(2)p/p62 (red). A magnified view of *dPRPS* mutant fat body is shown. Scale bar 100 μm. Graphs show quantification of Ref(2)p/p62 under fed conditions. Error bar indicate SEM from triplicated three independent experiments (n = 125 per experiment). Statistical testing in 4A-B were performed using One-way ANOVA where ns = p>0.05; * = p ≤ 0.05; *** = p ≤ 0.001; **** = p≤ 0.0001. (C and D) Graphs show survival of control and *dPRPS* mutant flies expressing RNAi against *atg8a* (C) and *atg16* (D) via *lsp2-Gal4* under starved conditions. Error bar indicate SEM from triplicated three independent experiments (n = 25 per experiment). Statistical testing in 4C was measured using Log-Rank test as compared to control (p ≤ 0.05 Q165P, p≤0.01 Control; Atg8a^RNAi^, p ≤ 0.05 Q165P; Atg8a^RNAi^). Statistical testing in 4D was measured using Log-Rank test as compared to control (p ≤ 0.05 Q165P, p≤0.01 Control; Atg16^RNAi^, p≤0.01 Q165P; Atg16^RNAi^).

### *dPRPS* mutants have lysosomal dysfunction

The endosomal system plays a critical function during macroautophagy [29]. Autophagosomes are generated at the endoplasmic reticulum (ER) and undergo a series of fusion processes with various endolysosomal compartments and lysosomes [29]. To determine whether an obvious abnormality exist in the endolysosomal system of *dPRPS* adult mutant flies, we visualized the ER, early endosome, and lysosome using anti-Calnexin (S4A Fig), anti-Rab5 (S4B Fig), and GFP-tagged Lamp1 (GFP-Lamp1) (Fig 5A), respectively. Strikingly, while the anti-Calnexin and anti-Rab5 did not show obvious differences, GFP-Lamp1 revealed that the lysosomal compartment is almost undetectable in *dPRPS* mutant fat bodies (Fig 5A). Two additional molecular markers were used to monitor lysosome function: LysoTracker, a membrane-permeable dye marking acidic compartments such as the lysosome, and Magic Red, a substrate-based fluorescence marker of Cathepsin B [30]. Similar to what was observed with the GFP-Lamp1, signals from both LysoTracker and Magic Red were significantly diminished in *dPRPS*^*Q165P*^ and *dPRPS*^*R228W*^ fat bodies while present in control fat bodies (Fig 5B and 5C). Importantly, mitochondria were readily detected in both the control and *dPRPS* mutant fat bodies (S4C Fig), indicating that the lysosome is specifically affected in *dPRPS* mutants. We also treated *dPRPS* mutant flies with chloroquine, a known inhibitor of lysosome function (Fig 5D) [31]. *dPRPS*^*Q165P*^ and *dPRPS*^*R228W*^ flies are more sensitive to chloroquine than control flies, indicating that lysosome function is indeed compromised in the mutant flies. Overall, our results indicate that the dPRPS is required for lysosome homeostasis and possibly contributes to the autophagy defect described in Fig 4.

**Fig 5:** *dPRPS* mutants have lysosomal dysfunction. (A) GFP-tagged Lamp1 (GFP-Lamp1) was used as a molecular marker to visualize the lysosome. A magnified view of the indicated area is also presented below. Scale bar: 100 μm. (B-C) Adult fat bodies of control and *dPRPS* mutant flies under fed conditions are stained with lysotracker (lyso) (B) or Magic red (MR) (C) to monitor lysosomal activity and active lysosomal cathepsins respectively. They are also stained with DAPI to visualize nuclei (blue). A magnified view of the indicated area (white box) is presented below. Scale bar: 85 μm. (A-C) Graphs showing quantification of GFP-Lamp1 (A), lysotracker (B) and Magic Red (C) puncta are presented. Error bar indicate SEM from triplicated three independent experiments (n = 250 per experiment). Statistical testing in 5A-C were performed using One-way ANOVA where ns = p>0.05; *** = p ≤ 0.001; **** = p≤ 0.0001. (D) Control and *dPRPS* mutant flies were treated with chloroquine under fed conditions. The graph showing their survival is shown. Error bar indicate SEM from triplicated three independent experiments (n = 25 per experiment). Chloroquine treatment decreases the lifespan of *dPRPS*^*Q165P*^ and *dPRPS*^*R228W*^ flies (p ≤ 0.001 for both genotypes, Log-Rank test compared to control (Control + PBS).

### Role of purine metabolism in *dPRPS-*associated dysfunction

To identify critical metabolic pathways contributing to the *dPRPS* mutant phenotypes, key enzymes in purine and pyrimidine biosynthetic pathways were knocked down in the fat body. Among the genes tested, adenylosuccinate synthase (*dAdS*) depletion reduced the LysoTracker signals, recapitulating the effect of *dPRPS* knockdown (Fig 6A). Moreover, fat body-specific depletion of *dAdS* or *dPRPS* resulted in an increased sensitivity to starvation, similar to what was observed in *dPRPS*^*Q165P*^ and *dPRPS*^*R228W*^ flies (Fig 6B). Importantly, depletion of an E2F-target important for dNTP synthesis, ribonucleotide reductase small subunit (*dRNRs*), had no effect, indicating the effect of *dAdS* knockdown is specific (Fig 6A and 6B). *dAdS* is a crucial enzyme in purine biosynthesis that converts Inosine monophosphate (IMP) to Adenylossucinate, which eventually becomes Adenosine monophosphate (AMP). Interestingly, S-adenosylmethionine (SAM), which can be converted to AMP and replenish purine nucleotides independently of PRPP, is given to patients with Arts syndrome hoping to restore a deficiency caused by PRPS dysfunction [32]. To determine if SAM treatment can have an effect on dPRPS-associated phenotypes, we fed *dPRPS*^*Q165P*^ and *dPRPS*^*R228W*^ flies with a sub-lethal dosage of SAM throughout the larval stage and determined its effect in adult flies. We also fed the mutants with a sub-lethal dosage of PRPP, the direct product of a PRPS-catalyzed reaction. Strikingly, SAM treatment partially and PRPP treatment virtually rescued the increased sensitivity of *dPRPS*^*Q165P*^ and *dPRPS*^*R228W*^ flies (Fig 6C and S5B Fig). Moreover, analysis of the adult fat body revealed that SAM or PRPP treatment partially restored LysoTracker signals, explaining why they can rescue the increased sensitivity of *dPRPS* mutant flies to starvation (Fig 6D and S5C Fig). Importantly, while PRPP treatment also suppressed the accumulation of Ref(2)p/p62 puncta in *dPRPS* mutant fat bodies, SAM treatment failed to do so (Fig 6E and S5C Fig). This suggests that PRPP-dependent metabolic pathways other than purine biosynthesis may be critical for the autophagy defect and are required to fully restore the deficiency caused by dPRPS dysfunction. Furthermore, this likely explains why SAM treatment cannot fully rescue the increased sensitivity of *dPRPS* mutant flies to starvation. We therefore concluded that the phenotype observed in *dPRPS*^*Q165P*^ and *dPRPS*^*R228W*^ flies are contributed by a deficiency in purine metabolism.

**Fig 6:** Role of purine metabolism in *dPRPS-*associated dysfunction. (A) Adult fat bodies of control and flies expressing RNAi against *dPRPS*, *dADS* and *dRNRs* via *lsp2-Gal4* stained with lysotracker. DAPI is used to visualize nuclei. Scale bar: 100 μm. The efficiency of the RNAi was determined by RT-qPCR (S5A Fig). (B) Graphs showing survival of flies expressing RNAi against *dPRPS*, *dADS* and *dRNRs* via *lsp2-Gal4* under starvation Error bar indicate SEM from triplicated three independent experiments (n = 25 per experiment). Statistical significance was measured using Log-Rank test as compared to control (p ≤ 0.01 *dPRPS*, p ≤ 0.01 *dADS*, and p>0.05 *dRNRS*). (C) Under complete starvation, control and *dPRPS*^*Q165P*^ mutant flies are treated with either PBS or 30mM of PRPP or SAM. The graph showing their survival is presented. Error bar indicate SEM from triplicated three independent experiments (n = 25 per experiment). Statistical significance was measured using a Log-Rank test compared to control (Control + PBS). p>0.05 Control + PRPP, p>0.05 Control + SAM, p ≤ 0.001 Q165P+PBS, p ≤ 0.01 Q165P+PRPP, p ≤ 0.01 Q165P + SAM. (D-E) Adult fat bodies of control and *dPRPS*^*Q165P*^ fat bodies fed with PBS, PRPP or SAM stained with lysotracker (D) and Ref(2)p/p62 (E). DAPI is used to visualize nuclei. Scale bar: 70 μm. Graphs showing quantification of lysotracker (D) and Ref(2)p/p62 (E) puncta upon PRPP or SAM treatment are presented. Error bar indicate SEM from triplicated three independent experiments (n = 200 per experiment). Statistical testing in 6D-E were performed using One-way ANOVA where ns = p>0.5; **** = p≤ 0.0001.

### *dPRPS* plays a critical function during cellular response to oxidative stress

Autophagy and thus proper lysosome function are needed to protect cells against oxidative stress by removing damaged proteins and organelles [25]. Interestingly, *dPRPS* was identified as one of the transcripts whose expression is induced by oxidative stress [13]. While the *dPRPS* transcript level is unchanged upon starvation, it is upregulated in response to paraquat (PQT) treatment, a Parkinsonian toxin that can induce oxidative stress (S6A Fig). We utilized the *dPRPS GFP-trap* allele to monitor dPRPS expression in specific tissues and noted that GFP expression is correspondingly increased in the ovary of PQT-treated flies (Fig 7A upper panel). However, in the fat body where the basal expression level of the dPRPS is high, PQT treatment did not have any effect (Fig 7A lower panel). Nevertheless, our results indicate that dPRPS expression is regulated by the cellular level of reactive oxygen species (ROS) and suggests a critical function during oxidative stress. Supporting this notion, we observed that *dPRPS*^*Q165P*^ and *dPRPS*^*R228W*^ fat bodies have higher levels of ROS measured by a fluorescent marker a 2',7'-dichlorodihydrofluorescein diacetate (H2DCFDA) (Fig 7B). This observation and its role in autophagy/lysosome led us to hypothesize that dPRPS is required for protection against oxidative stress. Thus, we examined the survival of *dPRPS*^*Q165P*^ and *dPRPS*^*R228W*^ flies treated with PQT (Fig 7C) and hydrogen peroxide (Fig 7D). Strikingly, *dPRPS* mutants died faster than control flies when treated with each compound, demonstrating their hypersensitivity to oxidative stress. We next tested whether the hypersensitivity of *dPRPS* mutants to oxidative stress contributes to their susceptibility to starvation. Control, *dPRPS*^*Q165P*^ and *dPRPS*^*R228W*^ flies were fed with an antioxidant NAC, and its effect on survival upon starvation was determined. While NAC supplementation had little to no effect on control flies, the survival of *dPRPS* mutants were partially rescued (Fig 7E), suggesting that oxidative stress contributes to the hypersensitivity of *dPRPS*^*Q165P*^ and *dPRPS*^*R228W*^ flies to starvation. Taken together, these results suggest that dPRPS is a ROS-regulated gene whose function is critical for cellular response to oxidative stress.

**Fig 7:** dPRPS plays a critical function during cellular response to oxidative stress. (A) Ovaries (upper panel) or fat bodies (lower panel) of adult *dPRPS GFP-trap* flies fed with PBS or PQT are immunostained for GFP (green) and DAPI (blue). (B) Adult fat bodies of control and *dPRPS* mutants are stained with H2DCFDA to measure the cellular ROS. Scale bar 50 μm. (C-E) Control and *dPRPS* mutant flies were treated with PBS, PQT (C) or hydrogen peroxide (D) under fed conditions. The graph showing their survival is shown. Error bar indicate SEM from triplicated three independent experiments (n = 25 per experiment). Paraquat treatment decreases the lifespan of *dPRPS*^*Q165P*^ and *dPRPS*^*R228W*^ flies (p≤0.01 for both genotypes, Log-Rank test compared to control (Control + PQT). Hydrogen peroxide treatment likewise decreases the lifespan *dPRPS*^*Q165P*^ and *dPRPS*^*R228W*^ flies (p ≤ 0.05 and p≤0.01, Log-Rank test compared to control (Control + H_2_O_2_). (E) Control and *dPRPS* mutant flies are treated with either PBS or NAC. The graph showing their survival upon starvation is presented. Error bar indicate SEM from triplicated three independent experiments (n = 35 per experiment). Statistical significance was measured using Log-Rank test compared to control (Control + PBS) (p ≤ 0.05 Q165P+PBS, p ≤ 0.05 R228W+PBS, p>0.05 Control + NAC, p≤0.01 Q165P+NAC, p ≤ 0.05 R228W+NAC).

### Patient-derived dPRPS mutations affect the nervous system

Given that the *dPRPS* mutant alleles are derived from Arts syndrome patients, we next investigated whether lipid mobilization, autophagy, and lysosome function are affected in the nervous system. A previous study has demonstrated that an accumulation of lipid droplets in surrounding glial cells of photoreceptor units in the adult eye is a common feature of *Drosophila* models of neurodegeneration [33]. We examined if a similar phenotype could be observed in *dPRPS*^*Q165P*^ and *dPRPS*^*R228W*^ flies. Indeed, we observed that lipid droplets accumulate in *dPRPS*^*Q165P*^ and *dPRPS*^*R228W*^ pupal eyes but not in control (Fig 8A). Additionally, mutations affecting autophagy in *Drosophila* often result in the accumulation of protein aggregates in the brain, caused by a failure to turnover damaged cytosolic proteins [34]. Since locomotive defects are observable in *dPRPS*^*Q165P*^ and *dPRPS*^*R228W*^ mutants as early as three days after eclosion (Fig 2E), we examined adult brains of three-day old control and *dPRPS* mutant flies. Anti-Ubi immunostaining (Fig 8B) and immunoblot (Fig 8C) revealed that *dPRPS*^*Q165P*^ and *dPRPS*^*R228W*^ have a higher level of ubiquitinated protein, suggesting that dPRPS function is required for proper clearance of damaged proteins. Notably, immunostaining resulted in a more striking difference than immunoblot. This is likely due to the formation of protein aggregates within the cell that amplifies the signal intensity. To better determine the role of PRPS in the nervous system, we depleted dPRPS in the nervous system using a pan-neuronal Gal4 driver, *ELAV-Gal4*. This was sufficient to produce accumulation of protein aggregates in the brain (Fig 8D) and to result in climbing defects (Fig 8E) while muscle-specific depletion had no effect (Fig 8F). Overall, these data suggest that the autophagy and lysosome defects, caused by the patient-derived PRPS mutations, affects the nervous system and provide a possible mechanism by which PRPS dysfunction contributes to neuropathogenesis.

**Fig 8:** *dPRPS* mutations affect the nervous system. (A) Pupal eye discs at 42 hours after pupa formation from control and dPRPS mutant flies stained with LipidTOX are shown. (B) 3-day old adult brains of control and *dPRPS* mutants are shown. An anti-Ubiquitin is used to visualize protein aggregates in the brain. Anti-Fasciclin (FasII) is used to visualize mushroom body neurons. Scale bar: 100 μm. (C) An immunoblot showing the level of ubiquitinated proteins in *dPRPS* mutant fly heads is presented. α-tubulin is used as a loading control. (D) 3-day old adult brains of control and flies expressing an RNAi against *dPRPS* via *ELAV-Gal4* (ELAV>) are stained with anti-ubiquitin and anti-FasII. Scale bar: 100 μm. (E-F) Climbing ability of flies expressing RNAi against *dPRPS* via *ELAV-Gal4* (E) and *Mef2-Gal4* (F) Statistical testing in 8E was performed using One-way ANOVA comparison to control at endpoint (t = 120 sec), p = 0.2484; ** = p ≤ 0.01.

## Discussion

In this study, we have established a Drosophila model of a PRPS-dependent neurological disorder. Using CRISPR/Cas9, mutations found in Arts syndrome patients were introduced to the only member of Drosophila PRPS. We uncovered that *dPRPS* is required for proper lipid mobilization, autophagy induction, lysosome function, and cellular response to ROS. Importantly, PRPS-dependent processes affect the nervous system, providing a possible mechanism by which PRPS dysfunction contributes to PRPS-associated neuropathology.

PRPS is a critical enzyme in nucleotide biosynthesis responsible for producing PRPP which is the five-carbon sugar subunit of nucleotides. Recent studies have shown that mammalian PRPS1 and 2 are regulated by genes and pathways that govern growth and proliferation such as Myc and AMPK [5, 12]. These studies demonstrated that PRPS is a key enzyme that couples metabolic demand to nucleotide production. It is unclear if dPRPS in Drosophila is regulated in a similar manner. However, our data showing that dPRPS is a Cic- and RBF1-regulated gene (Fig 1) and is required for Ras-induced hyperplastic overgrowth (Fig 2C), suggest its vital role in nucleotide metabolism downstream of signals controlling proliferation. Moreover, we found evidence indicating that PRPS expression is controlled by cellular level of ROS (Fig 7A and S6A Fig). It is probable that PRPS couples various environmental cues, including developmental signals, to regulate the rate of nucleotide synthesis. Importantly, we showed that dPRPS is critical for cellular level of autophagy and lysosomal homeostasis. An interesting possibility is that dPRPS expression is regulated to set the cellular level of autophagy and lysosome. This may also explain why in the fat body, where the basal level of autophagy is high [21], dPRPS expression is developmentally upregulated (S3A Fig). Of note, dPRPS expression is not induced by starvation indicating that the basal level of dPRPS is important for starvation-induced autophagy (S6B Fig). However, it is possible that dPRPS activity is post-transcriptionally regulated upon energy deprivation similar to what was observed with mammalian PRPS [12].

Two independent models of Arts syndrome-derived mutations we established in this study, *dPRPS*^*Q165P*^ and *dPRPS*^*R228W*^, have profound defects in autophagy and lysosome function. Importantly, these defects can be recapitulated by PRPS depletion (Figs 6A and 8D) and transheterozygous between patient-derived *dPRPS* mutations and a deficiency line covering the *dPRPS* locus (S7A–S7C Fig). This indicates that the patient-derived mutations decrease PRPS function and may not result in a gain of aberrant activity. Given the high degree of sequence homology (S1A Fig) and its essential role in nucleotide metabolism [1], it is probable that patients with *PRPS1*-associated disorders have similar defects described in this study. However, we have yet to pinpoint exact molecular and cellular processes that are affected by dPRPS dysfunction. Our data herein suggest that defects in autophagy and lysosome homeostasis may be independently affected by dPRPS dysfunction. This is most evident when *dPRPS*^*Q165P*^ and *dPRPS*^*R228W*^ are treated with SAM. While PRPP can suppress both autophagy and lysosomal defects, SAM only partially improves lysosomal defects (Fig 6D and 6E). In addition, lysosomal dysfunction alone cannot fully explain the autophagy defect described in this study. A recent study demonstrated that acidification is not required for autophagosome-lysosome fusion [35]. The v-ATPase-deficient non-acidic lysosomes can still fuse with autophagosomes, causing Atg8 to accumulate in abnormally large vesicles. This is certainly not the phenotype observed in *dPRPS* mutant fat bodies, where no Atg8a-puncta were detectable and indicative of defective autophagosome formation (Fig 4). Notably, our observations using various molecular markers of the lysosome all indicate that lysosomes are scarce in *dPRPS*^*Q165P*^ and *dPRPS*^*R228W*^ (Fig 5). The Drosophila mutants of *MITF*, a transcription factor important for lysosome biogenesis and homeostasis, show a similar phenotype as described in this study [36]. Detailed analysis comparing *dPRPS* and *MITF* mutant flies may tell us the role of lysosome in dPRPS-associated defects.

Because PRPP, the product of PRPS (Fig 1A), is a precursor for purines, pyrimidines, as well as pyridines that are important for a wide range of metabolic processes, it is unclear which dPRPS-dependent metabolic changes cause autophagy and lysosomal defects. We are in the process of performing extensive metabolic profiling and genetic dissection of the dPRPS-dependent pathways to determine the exact relationship between nucleotide metabolism and the endolysosomal system. However, we suspect that crucial metabolites missing in dPRPS-deficient cells can be non-cell autonomously provided. When clones of cells expressing the same *dPRPS* RNAi construct used in Fig 6A are generated in the fat body, they failed to show any decrease in LysoTracker signals (S8 Fig). Since the same RNAi construct were able to decrease the LysoTracker signals when expressed in the entire tissue (Fig 6A), this is unlikely due to inefficient knockdown. We hypothesize that neighboring wild-type cells produce and provide missing metabolites and/or their precursors to the dPRPS-deficient cells. While the identity of the exact metabolite is unclear, our data indicate that SAM or PRPP can be non-cell autonomously provided to *dPRPS* mutant cells and suppress their defects (Fig 6C–6E).

Importantly, autophagy and lysosomal defects in *dPRPS* mutant larvae are not as pronounced as those observed in the adult flies (S7D and S7E Fig). It is possible that the difference in the feeding behavior and metabolic status of larvae compared to the adult may affect the overall consequence of PRPS dysfunction. Perhaps, constant intake of food during the larval stage can partly compensate for the PRPP deficiency in *dPRPS*^*Q165P*^ and *dPRPS*^*R228W*^ flies. Another factor that may explain why autophagy and lysosomal defects are more pronounced in adult flies is the role of macroautophagy during metamorphosis [37]. Several studies have demonstrated that remodelling of tissues such as fat body, salivary glands, and midgut during pupariation requires macroautophagy. PRPS dysfunction may lead to a failure of proper tissue remodelling during metamorphosis and the accumulative effects manifest in the adult stage. However, while macroautophagy is important for tissue remodelling, the Atg8 conjugation system is not essential for completion of pupariation. Null mutants of *atg7*, which functions as an E1-like enzyme for Atg8 and Atg12, complete metamorphosis despite an abnormal level of autophagy [38]. It is worth noting that the Atg8 conjugation machinery is not absolutely required for autophagy [39] and that our assays largely relies on GFP-Atg8a quantification. Further in-depth analysis such as transmission electron microscopy will determine the precise impact of *dPRPS*^*Q165P*^ and *dPRPS*^*R228W*^ mutations on autophagy and lysosome homeostasis.

Many studies have clearly demonstrated that defects in autophagy are involved in the pathologies of various nervous system disorders, such as Alzheimer’s, Parkinson’s and Huntington’s disease [40–42]. In addition, there is a growing body of evidence suggesting that lysosome-mediated processes are important for neuronal homeostasis [41]. Notably, missense mutations in *rab7*, a small GTPase that plays a regulatory role in the endolysosomal pathway and autophagy, were also identified in CMT, one of the neurological disorders associated with PRPS1 mutations [43]. To date, no treatment option is available for patients with PRPS1-associated neurological disorders, such as children with Arts syndrome [3, 44, 45]. Preliminary results from an open-label clinical trial revealed that dietary SAM supplementation stabilized neurodegenerative progression in one ARTS syndrome patient [16]. Likewise, in our study SAM treatment partially rescued the starvation sensitivity and lysosome dysfunction in *dPRPS*^*Q165P*^ and *dPRPS*^*R228W*^ flies (Fig 6C and 6D and S5B Fig). This suggests that the *dPRPS* mutants described in this study may be used to identify future therapies for *PRPS1*-associated disorders. Moreover, identifying the exact mechanism by which PRPS regulates autophagy and lysosome homeostasis may uncover a novel treatment option for *PRPS1*-associated neurological disorders.

## Materials and methods

### Fly stocks

*D*. *melanogaster* stock cultures were maintained at 25°C. All crosses were performed at 25°C with the exception of the *UAS-RAS*^*V12*^ crosses at 18°C. Following stocks were obtained from Bloomington stock center: *PRPS*^*Mi09551*^ (#53132), *PRPS*^*Mi09551*^-*GFP-trap* (#59305), *UAS-RAS*^*v12*^ (#4847), *UAS-Lipase* (#67142), *UAS-Atg8a* (#58309), *UAS-Atg16* (#58244), *Lsp2-Gal4* (#6357), *UAS-AdS*^*RNAi*^ (#33993), MEF2*-Gal4* (#27390), *ELAV-Gal4* (#8765) and the *BSC576* deficiency stock (#26827). The GFP-Atg8a and GFP-Lamp1 are from [46]. The *cic*^*Q474X*^ mutant allele used in this project, including the method of generating clones in the eye has been previously described in [14]. The *rbf1*^*cas21*^ allele that normally contains *rbf1* mutant clones in the eye, is used in this study. The full description of the allele can be found in [47]. To generate eyes mostly composed of *rbf1*^*cas21*^ mutant cells, an additional copy of eye-specific FLPs was introduced to the *rbf1*^*cas21*^ allele. The *UAS-PRPS*^*RNAi*^ construct used in this project was obtained from the Vienna Drosophila Resource Center (VDRC) (# 35112). The *UAS-RNRs*^*RNA*i^ construct used in this project was obtained from the Harvard Medical Centre Transgenic RNAi Project (TRiP).

*dPRPS*^*Q165P*^ and *dPRPS*^*R228W*^ mutants were generated through homology-directed protocol as previously described in [48]. Positive CRISPR lines were screened through T7 Endonuclease I assay following the manufacturer's instructions (NEB MO302S) and confirmed through sequencing their genomic DNA (S2A Fig). To ensure that the control used in this study is within the same genetic background as the CRISPR generated mutants, an allele that does not contain the intended mutation was selected during the screening process. This control allele is used for starvation assays, feeding treatments, ATP determination, triglyceride quantification, immunofluorescence staining, immunoblot, developmental tracking, lifespan, and climbing assays. Other genotypes used as control are specified otherwise.

Donor DNA for *dPRPS*^*Q165P*^: TCCTTTGCATCTCTTTCTACGCTGGCCAATGCACAGAGTCGTGCGCCCATCTCGGCCAAATTGGTGGCCAACATGCTGTCCGTTGCTGGAGCGGATCACATCATCACCATGGATCTGCACGCCTCACCGATTCAGGTAAGTCAGCCCATCAACAACATTTGTATATTTATCTTTGATATTAGAGTGATTTCTTATCGTGC

Donor DNA for *dPRPS*^*R228W*^: TGCGTAATAGATTAATAATGCTATTAATATTTCACTTTAAGTGTCACCTCAATTGCCGATCGACTGAACGTGGAGTTCGCTCTGATACACAAGGAGTGGAGAAGGCCAACGAAGTGGCCTCTATGGTACTGGTGGGTGATGTCAAGGACAAGATTGCCATTCTGGTCGATGACATGGCCGACACATGCGGCACCATTGTG

Guide RNA (gRNA) as follows:

*dPRPS*^*Q165P*^ forward: GTCGCCAACATGCTGTCCGTTGC

*dPRPS*^*Q165P*^ reverse: AAACGCAACGGACAGCATGTTGGC

*dPRPS*^*R228W*^ forward: GTCGCGCAAGAAGGCCAACGAA

*dPRPS*^*R228W*^ reverse: AAACCTTCGTTGGCCTTCTTGCGC

### Starvation assay

For each genotype, triplicate batches of 25 female flies (2–3 days old) were transferred to vials of either normal cornmeal medium (fed) or water supply only (1% agarose in H_2_O (starved)). Survival rates were determined by counting the number of dead flies diagnosed by lack of a sit-up response every 12–14 hours. Triplicate sets were performed.

### NAC, SAM and PRPP treatment

Eggs were laid in cornmeal medium treated with PBS, 10mg/mL of NAC (Sigma), 30mM of PRPP (Sigma) or 30mM of SAM (NEB) to allow larvae to develop in the presence of each compound. Triplicate batches of 25 female flies, for SAM or PRPP, or 35 female flies, for NAC, were then collected and kept in the same media until they are 2–3 days old. Starvation assays were performed as described above.

### Chloroquine, paraquat and hydrogen peroxide treatment

Triplicate batches of 25 2–3 day old females were transferred to cornmeal medium treated with 20mM of chloroquine (Sigma), 30mM of paraquat (Sigma) or 1% hydrogen peroxide (Sigma). Survival rates were determined by counting the number of dead flies diagnosed by lack of a sit-up response every 12–14 hours. Triplicate sets were performed.

### RNA extraction and cDNA synthesis

RNA was extracted using the RNeasy Mini Kit (Qiagen) according to manufacture specifications. RNA was collected from whole *yw* flies (n = 5) for the measurement of *dPRPS* transcript levels in adult females fed normal yeast medium supplemented with 1X phosphate buffered saline (PBS), N-acetyl cysteine (NAC), or paraquat (24 hours). 500 ng of RNA was reverse transcribed using the DyNamo cDNA synthesis kit (ThermoScientific).

### Reverse transcriptase quantitative PCR

Reverse transcriptase qPCR (RT-qPCR) experiments were done using DyNAmo Flash SYBR Green qPCR kit (ThermoScientific) according to the manufacture specifications. Threshold cycle (CT) was determined using the Bio-Rad CFX Manager software. *rp49* and *β-tubulin* were both used for normalization. Each primer reaction was performed in triplicates and the three biological replicates were averaged. Primers were designed using Primer3 (*Whitehead Institute for Biomedical Research Primer3 shareware*, Frodo.wi.mit.edu/Primer3). The following primers were used for qPCR reactions:

*β-tubulin* forward: ACATCCCGCCCCGTGGTC

*β-tubulin* reverse: AGAAAGCCTTGCGCCTGAACATAG

*dPRPS Exon4* forward: CTTAGCAAGGGGTGATTTGG

*dPRPS Exon4* reverse: CCTTGATCCACTTGAGTACC

*dPRPS-E1-E3* forward: TTCAGCAACTTGGAGACCTG

*dPRPS-E1-E3* reverse: CCATGGTGATGATGTGATCCD

*dRNRs* forward: *CGTCCAAGGAAAACATTGCTG*

*dRNRs* reverse: TGGTGCTATCCGTCAGAATCTT

*dAdS* forward: CCGGCTTACTCCAGCAAGG

*dAdS* reverse: GGCCACAATCGACTTGAACTTTT

### ATP determination

Five female flies (2–3 days old) were homogenized in 100 *μ*l of 6 M guanidine-HCl in extraction buffer (100 mM Tris and 4 mM EDTA, pH 7.8) to inhibit ATPases. Homogenized samples were frozen in liquid nitrogen, followed by boiling for 5 minutes. Samples were centrifuged and diluted with extraction buffer followed by the addition of luminescent solution (Invitrogen). Luminescence was measured on a luminometer (Turner Biosystems). Relative ATP levels were normalized to the total protein concentration determined by Bradford assay.

### Colorimetric quantification of triglycerides (TAG)

Triglyceride levels were measured using a coupled colorimetric enzymatic triglyceride kit following manufacture instructions (Stanbio). 5 adult flies per genotype were used for each sample measurement in triplicates. Protein levels were measured in conjunction with TAG levels using Bradford assay (BioRad).

### LipidTox staining

For whole-mount staining of adult fat bodies (< 36 hours after eclosion), were dissected in 1X PBS and fixed with 4% formaldehyde in PBS for 20 minutes at room temperature. The fixed samples were then washed twice with 0.1% triton in 1X PBS (0.1% PBST) for 10 minutes following incubation in 1X DAPI in 0.1% PBST at room temperature for 15 minutes. After washing with 0.1% PBST, samples were incubated in 1:500 HCS LipidTOX Red Neutral Lipid Stain (ThermoFisher H34476). Samples were visualized within 2 hours by *Leica* SP8 point-scanning confocal system on a *Leica* DMI6000B inverted microscope (provided by the Cell Imaging Analysis Network (CIAN) in the Core Facility for Life Sciences at McGill University).

### LysoTracker, magic red and mitotracker staining

Adult fat bodies (2–3 days old) were dissected in 1X PBS and stained with either LysoTracker Red (1:1000, ThermoFisher L7528) or Magic Red (1:150, BioRad IT937) Mitotracker (1:300, ThermoFisher M7512) for 5, 15 and 30 minutes respectively. Samples were directly visualized using *Zeiss* Axio Imager fluorescent microscope.

### ROS detection

Adult fat bodies (2–3 days old) were dissected in Schneider’s Media and immediately incubated in 10 μm 5-(and-6)-carboxy-2′,7′-dichlorodihydrofluorescein diacetate, acetyl ester (CM-H2DCFDA, Molecular Probes, Invitrogen C6827) for 5 minutes. The samples were then washed twice with 0.1% triton in 1X PBS (0.1% PBST) for 10 minutes following incubation in 1X DAPI in 0.1% PBST at room temperature for 15 minutes. Samples were visualized within 30 minutes using *Zeiss* Axio Imager fluorescent microscope.

### Immunostaining

The following antibodies were used in this study: anti-Calnexin antibody (1:100, Abcam 75801), anti-Rab5 (1:100, Abcam 18211), anti-Fasciclin II (1:100, DHSB 528235), anti-Ref(2)p/p62 (1:100, Abcam 78440), anti-PH3 (1:100, Abcam 5176), anti-DCP1 (1:100, Cell Signalling 9578) and anti-GFP-FITC (1:200, Abcam 25052). Adult fat bodies were dissected in 1X PBS and fixed with 4% formaldehyde for 20 minutes. Fixed samples were washed twice with 0.3% PBST (0.3% Triton-X-100 in PBS) for 10 minutes. Next, samples were incubated with the indicated antibody. Fat body images were taken using *Zeiss* Axio Imager fluorescent microscope. Adult brain images were taken using *Leica* SP8 point-scanning confocal system on a *Leica* DMI6000B inverted microscope (provided by the Cell Imaging Analysis Network (CIAN) in the Core Facility for Life Sciences at McGill University).

### Analysis of lipid droplets and puncta in fat bodies

Fat bodies and lipid droplet size were analysed using *ImageJ* software. Quantification of puncta was performed with *ImageJ* using the particle intensity and 3D objects counter plugin [49].

### Climbing assay

Climbing tests were performed as previously described [20]. Briefly, 20 adult flies were transferred into a 250 mL glass graduated cylinder and gently tapped to the bottom of the cylinder. The number of flies reaching the 190 mL line (17.5 cm) of the 250 mL graduated cylinder was measured every ten seconds for two minute increments. Ten trials were performed for each genotype. Error bars indicate standard deviation from triplicated experiments.

### Chromatin immunoprecipitation (ChIP)- Quantitative PCR (qPCR)

ChIP-qPCR experiments were performed as previously described in [50]. Briefly, chromatin was collected from *w*^*1118*^ flies. Presented data are averages of triplicated ChIP experiments which consisted of experimental duplicates followed by quantitative real time PCR reactions. Presented data for target loci enrichment is represented by percentage of input chromatin not subjected to immunoprecipitation. All primers were designed by Primer 3 and primers used for ChIP-qPCR analyses are following:

1. *rnrS* forward: TGACAAGCTGGGAAGCTAAA
2. *rnrS* reverse: AAAATCAGGGCTGTCGAGTG
3. *trc8* forward: GGCTGTGACTTTGGGATGAA
4. *trc8* reverse: ATATCGCCCGTGGCTTTT
5. *act88F* forward: CCAACTCAAATCGCTTCGAG
6. *act88F* reverse: CGCACTCACACACCTTTTAG
7. *dPRPS P1* forward: AGAACCAATTGAAAGCGGCA
8. *dPRPS P1* reverse: TCCAAGGCCCCATAAGACTG
9. *dPRPS P3* forward: GATAGGGCTTCGGGGAAAGA
10. *dPRPS P3* reverse: TGGGTAGTATTAAGGGCGTATCT

### Scanning electron microscopy

Images were taken on FEI Quanta 450 Environmental Scanning Electron Microscope (FE-ESEM) located at the Facility for Electron Microscopy Research at McGill University.

### Immunoblot

All blots were blocked with 5% skim milk powder in 0.1% PBS-Tween20. To measure ubiquitinated protein levels, adult fly heads were collected from control and *dPRPS* mutants at day 3. Anti-Ubiquitin (1:1000, Invitrogen and Anti- β-tubulin (1:1000, DSHB) were used as primary antibodies followed by anti-mouse HRP (1:2000, GE Healthcare).

### Nail polish imprinting

Adult eye size was examined by using the nail polish imprinting technique as previously described [51]. Adult heads were covered in clear nail polish and dried at room temperature for 1 hour. The nail polish imprint was peeled off using tungsten needles and immediately mounted in 100% glycerol. Minimum of 5 adult heads were analyzed.

## Supporting information

S1 Fig *CG6767* encode the *Drosophila* ortholog of *phosphoribosyl pyrophosphate synthetase* (*dPRPS*). (A) Sequence alignment of human PRPS1, mouse PRPS1, and the only *Drosophila* PRPS ortholog coded by *CG6767* is shown. The *Drosophila* PRPS has 89% protein sequence identity to mammalian PRPS1. Red boxes indicate examples of conserved amino acids that are mutated in human patients with neurological disorders. (B) Schematic of the genomic region of *CG6767* is shown. The two publicly available insertional mutant alleles are marked by arrowheads. Insertions are in the *dPRPS* intron upstream of exon 2. The *Mi09551* allele has a splice acceptor site in the cassette that introduces stop codons downstream of exon 1. The *GFP-trap* allele contains an insertion that inserts the GFP coding sequences in frame at the same location as *Mi09551*. The *GFP-trap* allele produces an internally-tagged GFP-dPRPS fusion protein. (C) *dPRPS* transcript levels were measured by qRT-PCR of control *yw*, homozygous PRPS-Mi09551 and PRPS-MiGFP:trap second instar larvae. The primer pair used in qRT-PCR to bind and amplify exon 4. The error bars indicate standard error of the mean (SEM) from three biological replicates. Statistical testing was performed using One-way ANOVA where ns = p>0.5; *** = p ≤ 0.001. (D) The sizes of larvae at five days after egg laying (AEL) are compared. Control (*yw*), *Mi09551* heterozygote (*dPRPS*^*Mi551/+*^), *Mi09551* over a deficiency line (*dPRPS*^*Mi551/Df*^), *GFP-trap* heterozygote (*dPRPS*^*MiGFP/+*^), and *GFP-trap* over a deficiency line (*dPRPS*^*MiGFP/Df*^) are shown.
(TIF)

S2 Fig *dPRPS* mutant flies develop normally. (A) Genomic sequencing results of *dPRPS*^*Q165P*^ and *dPRPS*^*R228W*^ alleles. Two conserved amino acids shown in S1A Fig (red boxes) are edited and the changes in the codon (yellow boxes) are confirmed by sequencing (red letters). (B) Levels of *dPRPS* transcript were measured by qRT-PCR from control and *dPRPS*^*Q165P*^ and *dPRPS*^*R228W*^ third instar larvae. (3 biological replicates; mean values ± SEM are expressed relative to levels in control eye discs.) (C) Graph shows eclosion rate of control and *dPRPS* mutants. Days AEL: days after egg laying. Error bars indicate SEM from triplicated experiments (n = 100). (D) Representative images of control and *dPRPS* wings are shown. Scale bar: 0.5mm. Graphs show wing area. Error bars indicate SEM from ten individual flies. (E) Adult eyes of control and *dPRPS* mutant are pictured. Scale bar: 100 μm. Graph shows size of control and *dPRPS* mutant eyes. Error bars indicate SEM from five individual fly eyes. **(**F) Pupal eye discs 24 hrs after pupal formation are stained with pH3 marking mitotic cells. Discs overexpressing *Ras*^*V12*^ in control and *dPRPS*^*Q165P*^ backgrounds are presented. Scale bar: 100 μm. **(**G) Eye discs of *Ras*^*V12*^ overexpression in control and *dPRPS*^*Q165P*^ pupal eye discs 26 hrs after pupal formation stained with a cleaved form of a Drosophila caspase (Dcp1) marking apoptotic cells. Scale bar: 100 μm. Statistical testing in S2B-E were performed using One-way ANOVA where ns = p>0.5; * = p ≤ 0.05.
(TIF)

S3 Fig *dPRPS* is strongly expressed in the fat body. (A) Publically available transcript anatomical expression data of *CG6767* from *FlyAtlas* is shown (http://flyatlas.gla.ac.uk/FlyAtlas2/index.html?search=gene&gene=CG6767&idtype=cgnum#mobileTargetG). (B) Third instar larval fat bodies of control *yw* (upper) and *dPRPS GFP-trap* heterozygous (lower) immunostained for GFP are shown. (C) Graphs showing survival of control and *dPRPS* mutant adult flies under fed (left) and starved (right) are presented. Error bars indicate SEM from three independent triplicated experiments (n = 25). Starvation decreases the lifespan of *dPRPS*^*Q165P*^ and *dPRPS*^*R228W*^ flies (p ≤ 0.001 for both genotypes, Log-Rank test compared to control.
(TIF)

S4 Fig *dPRPS* mutants have functional mitochondria, endoplasmic reticulum and early endosome. (A—C) Adult fat bodies of control and *dPRPS*^*Q165P*^ flies under fed condition are stained with (A) anti-Calnexin, (B) anti-Rab5 or (C) mitotracker to visualize the endoplasmic reticulum, early endosome, and mitochondria respectively. They are also stained with DAPI to visualize nuclei (blue). Scale bar: 70 μm.
(TIF)

S5 Fig The role of purine metabolism in the *dPRPS^R228W^* mutant background. (A) RT-qPCR was performed to determine levels of knockdown of *dPRPS*, *dAdS* and *dRNRs*. (3 biological replicates; mean values ± SEM are expressed relative to levels in control fat bodies.) (B) Under complete starvation, control and *dPRPS*^*R228W*^ flies are treated with either PBS or 30mM of PRPP or SAM. The graph showing their survival is presented. Error bar indicate standard deviation from three independent triplicated experiments. Statistical significance was measured using a Log-Rank test compared to control (Control + PBS). p>0.05 Control + PRPP, p>0.05 Control + PBS, p ≤ 0.01 R228W+PBS, p ≤ 0.01 R228W+PRPP, p ≤ 0.01 R228W + SAM. (C) Adult fat bodies of *dPRPS*^*R228W*^ fed with PBS, PRPP or SAM stained with lysotracker (upper panel) and Ref(2)p/p62(lower panel). DAPI is used to visualize nuclei. Scale bar: 70 μm. Graphs showing quantification of lysotracker (left) and Ref(2)p/p62 (right) puncta upon PRPP or SAM treatment are presented. Error bar indicate SEM from triplicated three independent experiments (n = 200 per experiment). Statistical testing in S5A were performed using two-tailed t-tests where ns = p>0.5; *** = p ≤ 0.001. Statistical testing in S5C were performed using a One-way ANOVA where ns = p>0.5; *** = p ≤ 0.001; **** = p≤ 0.0001.
(TIF)

S6 Fig dPRPS expression is induced by oxidative stress. (A) *dPRPS* transcript levels were measured by quantitative RT-PCR. RNA is collected from control flies and flies fed with PBS (PBS) or paraquat (PQT). (3 biological replicates; mean values ± SEM are expressed relative to levels in control (oreR) fat bodies). Statistical testing was performed using One-way ANOVA where ns = p>0.5; ** = p ≤ 0.01; *** = p ≤ 0.001. (B) *dPRPS* transcript levels were measured by qRT-PCR. (3 biological replicates; mean values ± SEM are expressed relative to levels in control (oreR) fat bodies). Statistical testing was performed using two-tailed t-tests where ns = p>0.5.
(TIF)

S7 Fig Patient-derived *dPRPS* mutants are loss-of-function alleles and show reduced but detectable levels of autophagy and lysosome function at the larval stage. (A) Adult fat bodies of control and transheterozygous between *dPRPS*^*Q165P*^ and a deficiency line (Df) covering the *dPRPS* locus are stained with lysotracker and DAPI. Scale bar: 85 μm. (B) GFP-tagged Atg8a (GFP-Atg8a, green) was expressed via *lsp2-Gal4* to monitor autophagy under fed conditions in adult fat bodies of *dPRPS*^*Q165P*^/Df. DAPI is used to visualize nuclei (blue). Scale bar: 85 μm. (C) Graphs showing survival of control, *dPRPS*^*Q165P*^/Df and *dPRPS*^*R228W*^/Df adult flies during starvation are presented. Error bar indicate SEM from triplicated three independent experiments (n = 25 per experiment). *dPRPS*^*Q165P*^/Df and *dPRPS*^*R228W*^/Df flies have shorter lifespan than control (p ≤ 0.01 for both genotypes, Log-Rank test compared to control). (D) GFP-tagged Atg8a (GFP-Atg8a, green) was expressed via *lsp2-Gal4* to monitor autophagy under fed condition in larval fat bodies. DAPI is used to visualize nuclei (blue). Scale bar: 85 μm. Graph showing quantification of Atg8a-punctae are presented. (E) GFP-tagged Lamp1 (GFP-Lamp1, green) was expressed via *lsp2-Gal4* to monitor lysosome under fed condition in larval fat bodies. DAPI is used to visualize nuclei (blue). Scale bar: 85 μm. Graph showing quantification of GFP-Lamp1-punctae are presented. Error bar indicate SEM from triplicated three independent experiments (n = 180 per experiment). Statistical testing in S7D-E were performed using One-way ANOVA where * = p ≤ 0.05; *** = p ≤ 0.001; **** = p≤ 0.0001.
(TIF)

S8 Fig A hsFLP/FRT-mediate technique [52] was used to generate somatic clones expressing the same *dPRPS^RNAi^* construct used inFig 6A and 6B. The clones are positively marked by GFP. LysoTracker and DAPI are used to visualize lysosome and nucleus. *dPRPS* mutant clone cells are GFP-positive and outlined in yellow. Scale bar: 50 μm.
(TIF)
